The article "Effect of Kangfuxin Solution Fumigation Bath on Postoperative Patients with Hemorrhoid PPH and Influence on the Postoperative Complications" was retracted in 2023. Reasons: signs of a paper mill; compromised peer review; unreliable results or conclusions.

# Effect of Kangfuxin Solution Fumigation Bath on Postoperative Patients with Hemorrhoid PPH and Influence on the Postoperative Complications

**DOI:** 10.1155/2021/6473754

**Published:** 2021-09-08

**Authors:** Aiying Zeng, Gang Gu, Lin Deng

**Affiliations:** The Affiliated Nanhua Hospital, Department of Gastroenterology, Hengyang Medical College, University of South China, Hengyang, Hunan 421001, China

## Abstract

Surgery is now the main clinical treatment for hemorrhoids, and the procedure for prolapse and hemorrhoids (PPH) is the commonly used procedure. The key to evaluating the efficacy of surgery includes the quality of postoperative wound healing and the occurrence of complications, so it is especially important to enhance the postoperative rehabilitation of hemorrhoids. This study investigates the method of postoperative treatment with Kangfuxin solution fumigation bath to explore the role of this method in the efficacy of patients after hemorrhoid PHH surgery and its effect on postoperative complications. It will accumulate some relevant information to improve the efficacy of hemorrhoid surgery and postoperative complications and open new ideas for further postoperative rehabilitation of other diseases in the anal area. A total of 106 patients with hemorrhoids were included in this study, all of whom were treated with PHH surgery. After surgery, they were randomly divided into a control group treated with warm water sitz bath and an observation group treated with Kangfuxin solution fumigation bath, with 53 cases in each group. We observed all patients' postoperative pain, bleeding, and perianal edema on a daily basis after surgery; we recorded the time of wound healing and hospital stay. The maximum anal squeeze pressure (MASP), anal defecation diastole pressure (ADDP), anal resting pressure (ARP), and the length of the high-pressure zone (HPZ) were used as observation indicators to evaluate the anal function of the patients before and after treatment. The results of the evaluation of the efficacy of patients after the treatment period showed that the total effective rate of treatment in the observation group (92.45%) was significantly higher than that of the control group (77.36%). The postoperative recovery showed that the wound healing time, hospitalization time, pain, bleeding, and edema scores at 3 and 5 days after surgery were lower in the observation group than in the control group; MASP and ARP increased in both groups after treatment compared to before treatment, with more increase in the observation group. The results suggest that patients with hemorrhoids after PPH should pay attention to postoperative care and rehabilitation. It also reveals that the application of Kangfuxin solution fumigation treatment has a significant effect, which can effectively reduce the patient's wound healing and hospital stay, while improving the patient's anal function and reducing postoperative complications, and is worthy of clinical promotion and application.

## 1. Introduction

Hemorrhoids are one of the most common anorectal diseases that can be seen at any age and show a gradual increase in incidence with age [1]. Chronic constipation, alcohol abuse, consumption of irritating foods, and the sedentary lifestyle of the modern population are usually considered to be the main causes of hemorrhoids [2]. The anastomosis procedure for prolapse and hemorrhoids (PPH) uses the “PPH anastomosis” to cure hemorrhoids by circumferential excision of the prolapsed rectal mucosal band above the hemorrhoid [3]. It can preserve the normal physiological function of the anus to the greatest extent without removing the anal cushion and has the advantages of less trauma and faster recovery, so it can be rapidly promoted in clinical use [4].

However, due to the special anal site, postoperative defecation and medication changes can affect wound recovery as well as the healing effect, which can have a greater impact on patients' quality of life [5]. Therefore, effective anti-infection measures and enhanced postoperative rehabilitation after PPH for hemorrhoids are particularly important for wound healing and recovery and improving the quality of life of patients [6]. At present, Western medicine mainly focuses on symptomatic treatment in the treatment of complications after hemorrhoid surgery, and there is a lack of specific treatments that can significantly promote the recovery of complications after hemorrhoid surgery [7]. Chinese herbal fumigation is one of the more unique external treatment methods, which combines thermal effects and drugs on the treatment site to promote lymphatic reflux, improve blood circulation, relieve muscle spasm, and thus play a role in reducing pain and edema and promoting healing [8]. The main component of Kangfuxin solution is the extract of *Periplaneta americana*, which is a purely traditional Chinese medicine preparation with the effects of promoting blood circulation, nourishing yin fluid, and generating muscle [9]. In China, it is widely used in the treatment of stomach ulcer [10] and colitis [11] and has remarkable effects. In this study, we compared the clinical data of patients treated with different postoperative treatment modalities and investigated the efficacy of Kangfuxin solution fumigation bath in treating patients after PPH surgery for hemorrhoids and its effect on postoperative complications.

## 2. Materials and Methods

### 2.1. Materials

#### 2.1.1. Clinical Data

A total of 106 patients who underwent PPH surgery for hemorrhoids in our department from January 2019 to November 2019 were selected. There were 56 males and 50 females, aged from 21 to 58 years, with a mean age of (41.08 ± 8.27) years and a disease duration of 8 months to 12 years. 106 patients were randomly divided into a control group and an observation group of 53 patients each, in which the control group patients were treated with warm water sitz bath after surgery and the observation group patients were treated with Kangfuxin solution fumigation after surgery. There was no statistically significant difference between the two groups of patients in terms of baseline information such as gender, mean age, disease distribution, disease typing, condition, operative time, and intraoperative bleeding (*P* > 0.05, Table 1). The study was reviewed and approved by the hospital ethics committee, and the patients were informed and signed consent forms for the treatment protocol used in the study.

#### 2.1.2. Diagnostic Criteria [12]

1. Internal hemorrhoids: the main clinical manifestations are bleeding and prolapse, which can be complicated by thrombosis, impaction, strangulation, and defecation difficulties
2. External hemorrhoids: the main clinical manifestations are soft tissue masses in the anus, anal discomfort, itching or foreign body sensation, and pain if thrombosis and inflammation occur
3. Mixed hemorrhoids: the main clinical manifestations are the simultaneous presence of internal and external hemorrhoids, and in severe cases, the prolapse of circular hemorrhoids

#### 2.1.3. Inclusion Criteria

1. Patients who meet the diagnostic criteria
2. Patients who underwent hemorrhoid surgery for the first time
3. Nonscar or allergic constitution
4. No coagulation abnormalities
5. Patients in the age range of 20 to 60 years
6. Those who meet the internal hemorrhoid grade II or above [13]

#### 2.1.4. Exclusion Criteria

1. Combined with other anal diseases such as anal fissure, anal fistula, perianal abscess, rectal polyps
2. Patients with malignant tumors of the organism
3. People with infectious diseases
4. Pregnant women and women who are menstruating or breastfeeding
5. Patients who cannot cooperate with treatment
6. Patients in poor health with severe underlying medical conditions that preclude surgery

### 2.2. Methods

#### 2.2.1. Surgical Method

All patients underwent preoperative skin preparation after completing relevant preoperative examinations and confirming no significant abnormalities. Patients were instructed to fast and abstain from food and water for 6 hours before the operation; 0.9% sodium chloride solution (China Resources Shuanghe Pharmaceutical Co., Ltd.; approval number: H20056131) (500 ml) was used to clean the enema twice before the operation. The intramuscular injection of phenobarbital 0.1 g (Shanghai ShangPharma Xinya Pharmaceutical Co., Ltd.; approval number: H31020502) was used 30 minutes before surgery, while 1.0 g of cefathiamidine was injected intravenously (GuoPharm Zhijun (Shenzhen) Pharmaceutical Co., Ltd.; approval number: H20143010).

In both groups, the anesthesia was combined, spinal and epidural anesthesia, using levobupivacaine hydrochloride injection of 2 ml (Zhuhai Rundu Pharmaceutical Co., Ltd.; approval number: H20070023) at the L3-4 site; the surgical position was cystotomy in both groups. The anus was expanded with an anal canal dilator and the anal mirror was fixed. Insert the disposable tube-type hemorrhoid anastomat (Zhejiang Hai Sheng Medical Equipment Co., Ltd., China), pull appropriately with fingers and rotate the anastomosis clockwise at the same time to strike the anastomat, rotate the anastomosis counterclockwise one turn and remove it slowly after completing the anastomat, and then the anastomotic anastomosis and the integrity of the resected subrectal mucosa were inspected. All patients received conventional anti-infective treatment after operation. At the same time, they were given live combined bacillus subtilis and enterococcus faecium enteric-coated capsules (Beijing Hanmi Pharmaceutical Co., Ltd., approval number: S20030087) orally, with 0.25 g each time, 3 times daily to prevent diarrhea and constipation.

#### 2.2.2. Postoperative Rehabilitation Treatment

1. Control group: Warm water sitz bath was given for 10∼15 min after stool or in the morning and evening starting from the 1^st^ postoperative day, 2 times daily, and the treatment lasted for 5 days.
2. Observation group: Nebulized fumigation bath treatment with multifunctional perianal ultrasonic fumigation treatment instrument (Shanghai Hanfei Medical Devices Co., Ltd., China) was started on the 1^st^ postoperative day. 25 ml of Kangfuxin solution (Sichuan Good Doctor Panxi Pharmaceutical Co., Ltd.; approval number: Z51021834) and 200 ml of water were mixed and placed in the treatment instrument. The patient was helped to sit on the fumigation chair after placing a disposable isolation pad on the seat. After the patient sat on the fumigation chair, the nozzle was set to align with the anus and the mode of “cleaning-fumigation-heat therapy” was selected for treatment. The treatment was performed once a day for about 10–15 min each time and lasts for 5 days.

#### 2.2.3. Observation Indicators

Postoperative pain, bleeding, and perianal edema were observed daily in all patients after surgery, and the time of wound healing and hospital stay were recorded. The maximum anal squeeze pressure (MASP), anal defecation diastole pressure (ADDP), anal resting pressure (ARP), and the length of the high-pressure zone (HPZ) were measured before and after treatment in patients using ZGJ-D3 anal pressure detector (Shanghai Hanfei Medical Devices Co., Ltd., China) to assess anal function.

#### 2.2.4. Judgment Criteria

1. The criteria for determining the efficacy were as follows: Patients with hemorrhoids and symptoms disappeared were recognized as cured; patients with hemorrhoids disappeared and symptoms improved significantly were recognized as markedly effective; patients whose hemorrhoids disappear and whose symptoms are better than before were recognized as valid; patients with residual hemorrhoids or no relief of symptoms were considered invalid. Total effective rate = (number of cured cases + number of markedly effective cases)/total number of cases × 100%.
2. Pain scoring criteria: There were 4 levels in total, and the scoring range was 0∼3. A score of 0 indicated that the patient had no symptoms of pain; a score of 1 indicated that the symptoms of pain had no effect on the patient's work and life; a score of 2 indicated that the pain was unbearable and needed to be controlled with pain medication; and a score of 3 indicated that the pain had a serious effect on the patient's work and life.
3. Bleeding scoring criteria: There were 4 levels in total, and the scoring range was 0∼3. A score of 0 indicated that the patient had no symptoms of bleeding; a score of 1 indicated that blood was visible on toilet paper after stooling; a score of 2 indicated that blood was visible dripping during stooling; and a score of 3 indicated that visible jet-like bleeding was visible during stooling.
4. Edema scoring criteria: There were 4 levels in total, and the scoring range was 0∼3. A score of 0 meant that the patient had no symptoms of edema; a score of 1 meant that the area of edema was less than 25% perianal; a score of 2 meant that the area of edema was less than 50% of the perianal; and a score of 3 meant that the area of edema> 50% of the perianal.

### 2.3. Statistical Methods

SPSS 20.0 software was used for data processing, and GraphPad prism 8 was used to make statistical graphs. Measurement data were expressed as mean ± standard deviation ($\bar{x}$ ± *s*), the *t*-test was used for comparison between two groups, the rank-sum test was used for nonparametric test of grade data. Categorical information was expressed as (*n*, %), using the chi-square test. *P* < 0.05 was considered a statistically significant difference.

## 3. Results

### 3.1. Comparison of Clinical Efficacy

After 5 days of postoperative rehabilitation treatment, 21 cases (39.62%) in the control group were cured, 20 cases (37.74%) were markedly effective, 9 cases (16.98%) were valid, and 3 cases (5.66%) were invalid, with a total effective rate of 77.36%. In the observation group, 30 cases (56.60%) were cured, 19 cases (35.85%) were markedly effective, 3 cases (5.66%) were valid, and 1 case (1.89%) was invalid, with a total effective rate of 92.45%. The results of statistical analysis showed that the total effective rate of treatment in the observation group was significantly higher than that in the control group (*P* < 0.05, Figure 1), which suggested that the fumigation treatment with Kangfuxin solution had a positive effect on improving the efficacy of patients after PHH surgery for hemorrhoids.

### 3.2. Comparison of Wound Healing Time and Hospitalization Time

We observed and counted the postoperative recovery of patients in both groups. The mean wound healing time and the mean hospital stay in the control group were (9.28 ± 2.28) and (5.17 ± 1.43) days, respectively, while the mean wound healing time and the mean hospital stay in the observation group were (9.28 ± 2.28) and (5.17 ± 1.43) days, respectively. The mean wound healing time and mean hospital stay in the observation group were significantly lower than those in the control group (*P* < 0.05, Figure 2), suggesting that postoperative rehabilitation of PHH with Kangfuxin solution could promote the patient to recover as soon as possible.

### 3.3. Comparison of Anal Function before and after Treatment

There was no statistically significant difference between the MASP, ADDP, ARP, and the HPZ in the observation group and the control group at pretreatment (*P* > 0.05). The MASP, ADDP, ARP, and HPZ of both groups after treatment were significantly improved compared with those before treatment. There was no statistically significant difference in ADDP and HPZ after treatment between the two groups (*P* > 0.05), while MASP and ARP in the observation group were higher than those in the control group, and the difference was statistically significant (*P* < 0.05) (Figure 3). This has shown a positive effect on the improvement of anal function in postoperative hemorrhoid patients treated with Kangfuxin solution.

### 3.4. Comparison of the Improvement of Complications during Treatment

The pain, bleeding, and hematoma scores of the two groups at 1 day after surgery were all in a similar range, and the difference was not statistically significant (*P* < 0.05). The pain, bleeding, and edema scores of the two groups were significantly lower than those of the postoperative day 1 at 3 and 5 days after surgery, with the pain, bleeding, and edema scores of the observation group being lower than those of the control group at 3 and 5 days after surgery at the same time (*P* < 0.05, Figure 4). It has been shown that the use of Kangfuxin solution for fumigation treatment can effectively survive the relief of symptoms associated with patients after PHH surgery for hemorrhoids.

## 4. Discussion

PPH surgery for hemorrhoids is designed based on the theory of the inferior displacement of the anal cushion of internal hemorrhoids, and the severe prolapsed hemorrhoids are treated by a circular excision of the lower mucosa and submucosa of the rectum through a special instrument called the anastomosis. It has been widely used in clinical practice because of its advantages such as less trauma and faster recovery [14, 15].

Traditional Chinese medicine believes that hemorrhoids are divided into two categories. One is caused by Yang Huo because the patient likes to eat spicy food, resulting in the accumulation of heat in the intestines and stomach, poor excretion from below, and generating hemorrhoids. It has more serious symptoms of pain but is also accompanied by symptoms of red and swollen anus, hard stool, and red urine. The other type is caused by Yin Huo. Or, due to excessive worry, the vital energy is extremely weak and lax and wants to be removed from the lower part of the body but cannot be removed immediately, causing hemorrhoids to accumulate. These hemorrhoids are slightly painful and swollen, and they have a greater impact on the patient's spirit, who often has a blue and white face and lips and has difficulty sitting and lying down [16, 17]. The patients who underwent PPH surgery for hemorrhoids mostly have pathological characteristics such as mixed deficiency and stagnation of blood, so they often need to use drugs to invigorate blood and remove stasis and tonify the middle to improve the state of the body after surgery. Chinese herbal fumigation sitz bath is an important method to promote the recovery of patients after hemorrhoid surgery, and herbal fumigation can greatly increase the area of drug contact with perianal wounds. At the same time, drugs in the form of vaporization fully penetrate the surgical wound and can enhance the absorption of drugs [18]. The results of this study showed that the overall effective rate of patients in the observation group was higher than that of the control group. The ultrasonic fumigation bath treatment with Kangfuxin liquid fumigates the wound in the form of atomization and vaporization, and the full immersion of the drug can make the meridian of the surgical site unblocked, open the skin pores, and smooth the flow of Qi and blood, so as to achieve the effect of activating blood and swelling, relieving pain and hemorrhage [19]. The results of this study also showed that the time required for wound healing and hospitalization in the observation group was lower than that in the control group, which was closely related to the efficacy of the Kangfuxin solution in effectively improving local blood circulation and promoting edema reduction and wound healing [20]. The special location of the anus, injuries directly caused by surgery, postoperative perianal edema, direct stimulation of the wound by feces during defecation, patient tension during dressing changes, and spasm of the perianal muscles can all lead to postoperative wound infection and abnormal anal function in patients. Therefore, anti-infective treatment and care after PPH is particularly important to accelerate wound healing and restore normal anal function in patients [21]. The results of this study showed that the MASP and ARP in the observation group were higher than those in the control group in the posttreatment period, which was related to the polyol components and epithelial growth factors enriched in the Kangfuxin solution. These components were able to promote cell growth at the surgical site while enhancing the anti-inflammatory and anti-infective effects to promote the peeling off of necrotic tissue and improve the patient's anorectal kinetic index, thus restoring normal anal function [22].

After hemorrhoid surgery, patients often suffer from anal pain and discomfort due to local tissue damage around the anus, resulting in constipation due to fear of defecation. While constipation can aggravate anal edge edema, forming a vicious circle that delays wound healing and aggravates anal pain; thus, the treatment of postoperative complications of hemorrhoids should be based on the principles of meridian dredging and moving qi and blood to improve blood circulation at the patient's surgical site [23, 24]. The results of this study showed that the improvement of pain, bleeding, edema, and other complications in the observation group was better than that in the control group at 3 and 5 days after surgery, which indicated that the use of Kangfuxin solution with ultrasonic nebulizing bath was beneficial in reducing and improving the corresponding symptoms of patients. As a drug for postoperative rehabilitation of hemorrhoids, Kangfuxin solution has various advantages such as painless use, low toxic side effects, and low price. When fumigating with rehabilitation new liquid, it relies on drug volatilization and heat to act on the affected area to make the qi and blood flow in the affected area, thus achieving the effect of improving local blood circulation, reducing capillary permeability, and decreasing inflammatory exudation [25]. Sitz baths have a positive effect on improving the therapeutic effect of patients with hemorrhoids and improving postoperative pain and edema, but attention needs to be paid during the treatment process: (1) keep the medicinal water used for sitz baths at a more constant temperature to avoid the medicinal temperature being too high to cause local burns that aggravate pain or the medicinal temperature being too low for the medicinal effect to rise and reduce the therapeutic effect. (2) The time of each sitz bath is controlled within 10∼15 minutes to avoid too long time to cause or aggravate local edema.

## 5. Conclusion

In conclusion, patients after PPH surgery for hemorrhoids should pay attention to nursing care and rehabilitation treatment. The application of Kangfuxin solution fumigation treatment is effective, which can effectively reduce the wound healing and hospitalization time of patients, as well as improving the anal function of patients and reducing postoperative complications, and it is worthy of clinical promotion and application.

## Figures and Tables

**Figure 1:** Comparison of clinical efficacy between the two groups. Compared with the total effective rate of the control group, ^*∗*^*P* < 0.05.

**Figure 2:** Comparison of postoperative recovery in the two groups. (a) Comparison of the mean wound healing time. (b) Comparison of the average hospital stay. Compared with the control group, ^*∗*^*P* < 0.05.

**Figure 3:** Comparison of anal function between the two groups before and after treatment. (a) Comparison of mean MASP. (b) Comparison of mean ADDP. (c) Comparison of mean ARP. (d) Comparison of the mean HPZ length. Compared with the same group of pretreatment, ^∧^*P* < 0.05; compared with the control group at the same time, ^*∗*^*P* < 0.05.

**Figure 4:** Comparison of the improvement of complications at 1, 3, and 5 days postoperatively in the two groups. (a) Comparison of mean pain scores at different postoperative times. (b) Comparison of mean bleeding scores at different times after surgery. (c) Comparison of mean edema scores at different times postoperatively. Compared with 1 day postoperatively, ^#^*P* < 0.05; compared with the control group at the same time point, ^*∗*^*P* < 0.05.

**Table 1:** Comparison of baseline information between the two groups.

Information		Control group (*n* = 53)	Observation group (*n* = 53)	*P* value
Gender (*n*, %)	Male	27 (50.94)	29 (54.72)	0.697
	Female	26 (49.06)	24 (45.28)	
	<1 year	3 (5.66)	4 (7.55)	

Disease duration (*n*, %)	1∼5 years	30 (56.60)	32 (60.38)	0.828
	5∼10 years	14 (26.42)	13 (24.52)	
	≥10 years	6 (11.32)	4 (7.55)	

Disease typing (*n*, %)	Internal hemorrhoids	32 (60.38)	33 (62.26)	0.842
	Mixed hemorrhoid	21 (39.62)	20 (37.74)	

Internal hemorrhoid grading (*n*, %)	Grade II	17 (32.08)	20 (37.74)	0.551
	Grade III	28 (52.83)	26 (49.06)	
	Grade IV	8 (15.09)	7 (13.21)	

Age, mean (SD), years		40.51 ± 9.14	42.73 ± 8.54	0.224
Surgery time, mean (SD), min		38.26 ± 2.23	37.59 ± 2.51	0.149
Intraoperative bleeding, mean (SD), ml		6.42 ± 0.78	6.37 ± 0.63	0.717

## Data Availability

The data used in the current study are available from the corresponding author on reasonable request.
